# Depletion of CD4^+^ CD25^+^ Regulatory T Cells Promotes CCL21-Mediated Antitumor Immunity

This article has been retracted.

**DOI:** 10.1371/journal.pone.0073952

**Published:** 2013-09-02

**Authors:** Shuang Zhou, Huihong Tao, Zhiwei Zhen, Haixia Chen, Guolin Chen, Yaoqin Yang

**Affiliations:** Department of Histology and Embryology, Tongji University School of Medicine, Shanghai, China; University of Nebraska Medical center, United States of America

## Abstract

CCL21 is known to attract dendritic cells (DCs) and T cells that may reverse tumor-mediated immune suppression. The massive infiltration of tumors by regulatory T cells (Tregs) prevents the development of a successful helper immune response. In this study, we investigated whether elimination of CD4^+^ CD25^+^ Tregs in the tumor microenvironment using anti-CD25 monoclonal antibodies (mAbs) was capable of enhancing CCL21-mediated antitumor immunity in a mouse hepatocellular carcinoma (HCC) model. We found that CCL21 in combination with anti-CD25 mAbs (PC61) resulted in improved antitumor efficacy and prolonged survival, not only inhibited tumor angiogenesis and cell proliferation, but also led to significant increases in the frequency of CD4^+^, CD8^+^ T cells and CD11c^+^ DCs within the tumor, coincident with marked induction of tumor-specific CD8^+^ cytotoxic T lymphocytes (CTLs) at the local tumor site. The intratumoral immune responses were accompanied by the enhanced elaboration of IL-12 and IFN-γ, but reduced release of the immunosuppressive mediators IL-10 and TGF-β1. The results indicated that depletion of Tregs in the tumor microenvironment could enhance CCL21-mediated antitumor immunity, and CCL21 combined with anti-CD25 mAbs may be a more effective immunotherapy to promote tumor rejection.

## Introduction

The induction of an effective antitumor immune response requires both antigen-presenting cells (APCs) and activated T cells. One might speculate that a stronger immune response could be achieved by attracting larger numbers of effector T cells and mature dendritic cells (DCs) to the tumor site. Increasing evidence shows that chemokines play an integral role in the initiation of a specific immune response [1,2].

CCL21, formerly known as secondary lymphoid tissue chemokine (SLC), is a CC chemokine that is capable of recruiting DCs, naive T cells and B cells via its specific receptor CCR7 (CC chemokine receptor type 7) found on these cell types [3–5]. Based on its expression pattern and that of its receptor, CCL21 could serve as a potent agent in cancer immunotherapy. Previous studies have demonstrated that CCL21 administered intratumorally elicits tumor rejection in murine models of established tumors [6,7]. We and others have also shown that vaccination with CCL21 modification is an effective strategy to stimulate antitumor immune responses in a mouse hepatocellular carcinoma (HCC) model [8–11]. The CCL21-mediated antitumor response is dependent on both CD4^+^ and CD8^+^ lymphocyte subsets, also accompanied by DCs infiltration [6]. However, it should be noted that CCL21 elicits a substantial infiltration of DCs and naive T cells into the tumor, as well as the naturally occurring regulatory T cells (Tregs) by means of CCR7 [12–14].

Tregs are thought to control key aspects of immunological tolerance to self-antigens. They are broadly identified as a small proportion of CD4^+^ T cells that highly express CD25 (IL-2Rα-chain) on their surface [15,16]. It has also been shown that Tregs specifically express Foxp3 (forkhead box P3) [17]. CD4^+^ CD25^+^ Tregs act in a regulatory capacity by suppressing the activation and function of other immunocytes, they can control immune responses induced by DCs in vivo [18], also prevent CD8^+^ T cell maturation by inhibiting CD4^+^ Th cells at tumor sites [19]. Tregs are present in high frequencies among tumor-infiltrating lymphocytes supposedly facilitating tumor development [20]. Thus, Tregs accumulate in the tumor microenvironment and inhibit antitumor immunity, presenting a major obstacle for developing effective and therapeutic cancer vaccines. This notion could explain anti-CD25 monoclonal antibodies (mAbs) treatment inducing tumor rejection in animal models [21,22].

A potential problem associated with the use of CD25-specific antibodies is the simultaneous depletion of conventional CD25^+^ effector T cells, whose loss may compromise the beneficial effect of depleting the Tregs [23]. Previous studies have indicated that treatment of mice with anti-CD25 mAbs is only beneficial within a limited time window, in the later time points anti-CD25 mAbs will not only deplete Tregs, but also affect the effector cells that are involved in tumor rejection [24–26]. It is undeniable that the beneficial effect of Tregs depletion in tumor regression is abrogated when CD4^+^ helper cells are also depleted. Therefore, a combination of anti-CD25 and vaccination may be necessary and provide an improved immunotherapeutic approach for tumors.

In this study, we performed a combination treatment of CCL21 and anti-CD25 mAbs (PC61) in a mouse HCC model. This approach attempts to attract mature host DCs and activated T cells at the tumor site, meanwhile, the suppressive effects of Tregs can be reduced. Our results suggested that CCL21-mediated antitumor immunity was strengthened when combined with anti-CD25 mAbs administration, characterized by increasing the frequency of tumor-specific CD8^+^ T cells and CD11c^+^ DCs, and enhancing the production of IL-12 and IFN-γ within the tumor, leading to improved antitumor efficacy.

## Materials and Methods

### Animals

C57BL/6J (H-2b) female mice, 6 to 8 weeks of age, were purchased from the Chinese Academy of Science and housed at the Animal Maintenance Facility of Tongji University. The protocol was approved by the Animal Ethics Committee of Tongji University. All animal experiments were performed under specific pathogen-free conditions in accordance with institutional guidelines.

### Tumor cell line

The murine Hepal-6 hepatocellular carcinoma cell line (CRL-1830) was from American Type Culture Collection (ATCC). Hepa1-6 cell line was transfected with pRRL-CMV lentiviral-luciferase vector to creat a stable luciferase expression clone selected by limited dilution. Cells (Luc-Hepa1-6) were propagated in RPMI 1640 supplemented with 10% heat-inactivated fetal calf serum (GIBCO-BRL), 0.1 mM nonessential amino acids, 1 µM sodium pyruvate, 2 mM fresh L-glutamine, 100 µg/ml streptomycin, 100 units/ml penicillin, 50 µg/ml gentamicin, and 0.5 µg/ml fungizone, and maintained at 37°C in humidified atmosphere containing 5% CO2 in air.

### Treatment of established tumors

A total of 3×10^6^ Luc-Hepal-6 cells diluted in 200 µl of serum-free RPMI 1640 medium were injected subcutaneously into the right flank of C57BL/6J mice to inoculate tumors. On day 8 after inoculation, tumor-bearing mice were randomly divided into different treatment groups as follows (n = 8 for each group): (1) control group, intraperitoneal (ip) injection with 0.5 mg normal rat IgG1 in 200 µl PBS; (2) CCL21 treatment group, subcutaneous (sc) injection with 0.5 µg recombinant murine CCL21 (PeproTech, Rocky Hill, NJ) in 50 µl PBS in the right flank based on the previous study [6]; (3) anti-CD25 treatment group, ip injection with 0.5 mg purified anti-CD25 mAbs (PC61) in 200 µl PBS as previously described [22,27]; (4) combination treatment group, sc injection with 0.5 µg CCL21 in 50 µl PBS and ip injection with 0.5 mg anti-CD25 mAbs in 200 µl PBS. Anti-CD25 mAbs for in vivo administration and rat IgG1 control antibodies were obtained from Accurate Chemical and Scientific Corporation (Westbury, NY). CCL21 injections were administered one time every other day for five times. The administration of anti-CD25 mAbs or control antibodies was performed by a single injection on day 8 after inoculation. Tumor sizes were monitored every other day for 9 days with Vernier calipers after the start of treatment. Tumor volume was calculated by the formula: *V* (in mm^3^) = 0.5(*ab* ^2^), where *a* is the long diameter and *b* is the short diameter. The mice were subjected to imaging on day 7 after the start of treatment. On day 9 after treatment initiation, mice in all groups were sacrificed. Tumors were removed and weights were determined. Survival curve analysis and the following experiments were respectively done in the independent treatment groups.

### Bioluminescence imaging in vivo

The bioluminescence imaging was performed using an animal imaging system (NightOWL LB 983 Molecular Imaging System, Berthold, Germany). For in vivo imaging, the mice received an ip injection of 150 mg/kg D-luciferin potassium salt (Caliper Life Sciences, USA) in 200 µl DPBS. After 5 minutes of luciferin injection, the mice were anesthetized via ip injection of pentobarbital (50 mg/kg). Each mouse was placed in a left lateral decubitus position and a digital grayscale animal image was acquired, followed by the acquisition and overlay of a pseudocolor image representing the spatial distribution of detected photons emerging from active luciferase within the animal. Photons emitted from specific regions were quantified using a IndiGo software (Berthold). Regions of interest (ROI) were drawn around the tumor sites and quantified as photon counts per second.

### Flow cytometry

The tumors were mechanically dissociated in cold filter-sterilized PBS-3% BSA and gently mashed through a 70-µm-pore-size nylon mesh to produce a single cell suspension. Samples were stained with Alexa 488-conjugated anti-mouse CD25 (eBioscience, USA). Subsequently, the cells were fixed and permeabilized followed by PE-conjugated anti-mouse Foxp3 (eBioscience). Isotype controls for each antibody were also included. For analysis of effector cells infiltration, samples from day 7 after treatment initiation were stained with FITC-conjugated antibodies to mouse CD4, CD8 and PE-conjugated anti-mouse CD11c (eBioscience). All the samples were acquired on a FACSCalibur (Becton Dickinson, USA) counting of 20,000 lymphocyte-sized events and analyzed with WinMDI 2.9 software. Total cell populations for CD4^+^, CD8^+^, CD25^+^ Foxp3^+^ T cells and CD11c^+^ DCs were calculated by multiplying the percentage of occurrence in a dot plot of a cell population by the total number of cells counted.

### Immunohistochemistry

Tumor tissues were fixed in periodate-lysine-paraformaldehyde (PLP), embedded in O.C.T (Sakura Finetek, USA), and cut into 10 µm sections. Then, the sections were stained with specific antibodies for analysis. Tregs within the progressive tumor were double-stained with FITC-CD4 and Cy3-Foxp3 antibody (eBioscience). Nuclei were counterstained with DAPI (Sigma, USA). Isotype-matched antibodies were used as a control. Microvessel density and CD8^+^ T cells in tumor tissues were detected with rat anti-mouse CD31 antibody (BD Pharmingen, USA) and rat anti-mouse CD8 (eBioscience), followed by HRP-conjugated rabbit anti-rat IgG (Invitrogen, USA) and DAB liquid substrate system (Sigma), respectively. According to the method of Weidner et al [28], the quantification of microvessel density (MVD) was assessed. Cell proliferation was performed on the frozen tumor sections with rat anti-mouse Ki-67 antibody (Biolegend, USA) followed by FITC-conjugated rabbit anti-rat IgG (Invitrogen). Results were expressed as the percentage of Ki-67 positive cells ± SEM per ×400 magnification. A total of ten ×400 fields were examined and counted from three tumors in each of the treatment groups. The Ki-67 proliferation index was calculated according to the following formula: the number of Ki-67 positive cells/total cell count ×100%.

### Western blot analysis

Tumor tissues were homogenized with lysis buffer (RIPA) (50 mM Tris–HCl, pH 7.4, 150 mM NaCl, 1 mM EDTA, 0.1% SDS, 1% Triton X-100, 1% sodium Deoxycholate, 1 mM PMSF, 10 mg/ml aprotinin, 10 mg/ml leupeptin) on ice. After centrifugation at 14,000 rpm at 4°C for 30 min, supernatants were collected and total protein concentrations were determined by BCA assay (Pierce, USA). Equal amounts of denatured proteins were loaded onto 10% SDS-PAGE gel and transferred on PVDF membrane (Millipore, USA). Membranes were blocked with 5% nonfat milk in TBST (1×TBS containing 0.1% Tween 20), and then incubated with primary antibodies to CCR7 and Foxp3 (eBioscience) overnight, After washing with TBST three times, HRP-conjugated secondary antibodies (KPL, USA) were bound and performed with chemiluminescence using SuperSignal West Pico substrate (Pierce). Band intensities were quantified using Band Leader software.

### Cytokine ELISA

Levels of intratumoral cytokines (IL-12, IFN-γ, IL-10, and TGF-β1) were determined using commercially available ELISA kits (eBioscience). Frozen tumor tissue samples from day 7 after treatment initiation were accurately weighed and placed in cold RIPA buffer at a ratio of 100 mg tissue per milliliter. Samples were homogenized and subjected to one round of freeze-thaw, sonicated for 10 min, and incubated at 4 °C for one hour. The final homogenates were centrifuged at 14,000 rpm at 4°C for 30 min. Tissue supernatants were used for cytokine determination following the manufacturer’s instruction and the data were expressed at pg/mg tumor tissue.

### Statistical analysis

Statistical significance was determined using one-way ANOVA or Student’s *t* test, as appropriate. *P < 0.05 was considered statistically significant, and ** *P* < 0.01 would be highly statistically significant.

## Results

### Accumulation of Tregs and different expression patterns of CCR7 and Foxp3 within the progressive tumor

To explain the importance of Tregs depletion, Tregs in the tumor site were double-stained with CD4 and Foxp3 antibodies. The expression patterns of CCR7 and Foxp3 within the progressive tumor were identified by western blot. The results showed that CD4^+^ Foxp3^+^ Tregs gradually accumulated in the tumor tissue of early-stage HCC on day 8 and 14 after Hepa1-6 sc inoculation (Figure 1A), CCR7 downregulation and Foxp3 upregulation in the development of HCC from day 8 to 29 were also verified (Figure 1B).

**Figure 1:** Accumulation of Tregs and different expression patterns of CCR7 and Foxp3 within the progressive tumors. (**A**) CD4^+^ Foxp3^+^ Tregs were increased in the tumor tissues of early-stage HCC on day 8 and 14 after Hepa1-6 subcutaneous inoculation. Serial 5-µm-thick cryostat sections were double-stained with CD4 (green) and Foxp3 (red) antibodies. Scale bar, 50 µm. (**B**) CCR7 downregulation and Foxp3 upregulation in the development of HCC from day 8 to 29 were verified by western blot. β-actin was used as an internal control. Protein levels were determined by densitometry analysis and were expressed as ratios to β-actin (below each blot). The ratio obtained from the first lane was set as 1. All data were representative of at least two independent experiments.

### Maximal inhibition of tumor growth by combination therapy of CCL21 and anti-CD25 mAbs

The effects of combination treatment on the growth of Hepa1-6 tumors were evaluated in tumor-bearing mice models. Schedule of experimental procedures was showed in Figure 2A. Although CCL21 and anti-CD25 alone also significantly inhibited tumor growth after treatment, the combination therapy of CCL21 and anti-CD25 mAbs resulted in a more robust inhibition of tumor development, and had the most significant delay in tumor growth as determined by tumor volume after treatment initiation (Figure 2D) and tumor weight on day 9 when treatment was stopped (Figure 2E). Bioluminescence imaging analysis of tumor on day 7 after the start of treatment confirmed the antitumor effects (Figure 2B and C). Similarly, the increased tumor growth inhibition in the combination therapy was translated into the prolonged survival according to the Kaplan-Meier analysis and the mice received the combination therapy remained 100% survival at the end of observation period (Figure 2F).

**Figure 2:** Schedule of experimental procedures and antitumor effects of combination therapy with CCL21 and anti-CD25 mAbs in HCC model. (**A**) Schematic representation of experiment protocol described in materials and methods. Animals were divided into four groups (n = 8 for each group). (**B**) Representative bioluminescence images of Luc-Hepa1-6 tumors on day 7 after the start of treatment. (**C**) Imaging analysis (photons per second) depicting the tumor volumes of mice using the IndiGo imaging analysis software (n = 5 for each group). (**D**) CCL21 combined with anti-CD25 mAbs treatment resulted in maximally inhibition of tumor growth. Tumor sizes were monitored on day 1 to 9 after treatment initiation (n = 8 for each group). (**E**) The combination treatment significantly reduced tumor weight. Tumor weights were measured on day 9 after treatment initiation when harvested (n = 8 for each group). (**F**) Survival curves were constructed in the independent treatment groups according to the Kaplan-Meier method (n = 8 for each group). *P < 0.05, **P < 0.01, compared with the control group.

### Depletion of Tregs by anti-CD25 mAbs in CCL21-treated mice

To determine whether ip injection of anti-CD25 mAbs (PC61) led to a selective loss of Tregs in CCL21-treated mice, the population of CD25^+^ Foxp3^+^ Tregs within the tumors was assessed by flow cytometry respectively on day 1 to 9 after treatment initiation. Representative percentages of CD25^+^ Foxp3^+^ Tregs were shown in density plots (Figure 3A). The results from all test and control mice were summarized and provided in a curve diagram (Figure 3B). On day 1 to 7 after treatment initiation, intratumoral CD25^+^ Foxp3^+^ Tregs percentages remained essentially constant at a significantly lower level (*P* < 0.01) in CCL21 combined with anti-CD25 treated mice, as well as anti-CD25 treatment group, whereas even 6-fold lower mumbers of cells compared with control group. But there was a linear increase (range 1% to 4.8%) in CCL21 treatment group. Notably, we used two different Alexa 488-anti-mouse CD25 mAbs (PC61 or 7D4) to get analogous detection results for Tregs depletion confirmation in mouse spleen after a single ip injection of 0.5 mg anti-CD25 mAbs (data not shown).

**Figure 3:** Depletion of Tregs by anti-CD25 mAbs in CCL21-treated mice. Respectively on day 1, 3, 5, 7, 9 after treatment initiation in the independent treatment groups, mice were sacrificed and tumors were harvested for quantification of CD25^+^ Foxp3^+^ Tregs. (**A**) Flow cytometry analysis for the population of CD25^+^ Foxp3^+^ Tregs within the tumors on day 1 to 9 after treatment initiation. Representative percentages of CD25^+^ Foxp3^+^ Tregs were shown in density plots. (**B**) A curve diagram was summarized for the results from all test and control mice (n = 3 for each group). *P < 0.05, **P < 0.01, compared with the control group. Similar results were obtained in three independent experiments.

### Dynamic changes of CCR7 and Foxp3 expression after combination treatment

The chemotaxis effect of CCL21 can be measured by the level of intratumoral CCR7 expression, and depletion of Tregs can be defined by Foxp3 expression. The results demonstrated that coadministration of CCL21 with anti-CD25 mAbs resulted in dynamic changes of CCR7 and Foxp3 expression, upregulation of CCR7 and inhibition of Foxp3 expression on day 1 to 7 after treatment initiation (Figure 4).

**Figure 4:** Dynamic changes of CCR7 and Foxp3 expression after combination treatment. CCR7 and Foxp3 expressions in tumor tissue lysates on day 1 to 9 after treatment initiation were determined by western blot. β-actin was used as a an internal control. Protein levels were determined by densitometry analysis and were expressed as ratios to β-actin (below each blot). The ratio obtained from the first lane was set as 1. All data were representative of at least two independent experiments.

### Inhibition of tumor angiogenesis and cell proliferation

To estimate angiogenesis within the tumor tissue, microvessel counts were determined by immunohistochemical staining for CD31. The combination therapy resulted in a more obvious inhibition of the angiogenesis in tumors compared with the control and monotherapy groups. The average number of microvessels per high-power field from the section on day 7 after treatment initiation was highly statistically significant in the combination group (*P* < 0.01, Figure 5A and B). Immunohistochemical analysis of cell proliferation was performed on the frozen tumor sections on day 7 after treatment initiation with Ki-67 antibody. The Ki-67 proliferation index was calculated and showed a significant suppression in CCL21 treatment groups, which was 6-fold decrease in the combination group compared with the control group (*P* < 0.01, Figure 5A and C).

**Figure 5:** Inhibition of angiogenesis and proliferation within the tumors after combination treatment. (**A**) Representative images of CD31 positive microvessels and Ki-67 positive cells in tumor tissues on day 7 after treatment initiation estimated by immunohistochemical staining. Scale bar, 100 and 50 µm. (**B**) and (**C**) Microvessel density and percentage of Ki-67 positive cells were determined by counting the number of the positive staining per high-power field in the section, as described in “Materials and Methods”. *P < 0.05, **P < 0.01, compared with the control group.

### Enhancement of the frequency of CD4^+^, CD8^+^ T cells and CD11c^+^ DCs at the tumor site after combination treatment

To quantify the tumor-infiltrating CD4^+^, CD8^+^ T cells and CD11c^+^ DCs, the tumor samples on day 7 after treatment initiation, a representative time-point for Tregs depletion and tumor growth inhibition, were analyzed by flow cytometry. The results indicated that sc injection of CCL21 could increase the infiltration of CD4^+^, CD8^+^ and CD11c^+^ effector cells at the tumor site. Compared with the control group, there were significant increases in the frequency of CD4^+^ T cells in CCL21 treatment group or combination treatment group. Despite a small proportion loss of CD4^+^ T cells by anti-CD25 mAbs in the combination treatment group, there were significantly more infiltrating CD8^+^ T cells and CD11c^+^ DCs into the tumor (*P* < 0.01, Figure 6B), especially marked induction of tumor-specific CD8^+^ cytotoxic T lymphocytes (CTLs) at the local tumor site (Figure 6A).

**Figure 6:** The increased frequency of CD4^+^, CD8^+^ T cells and CD11c^+^ DCs at the tumor site after combination treatment. The tumor samples on day 7 after treatment initiation were assayed (n = 3 for each group). (**A**) Immunohistochemical analysis showed that marked infiltration of tumor-specific CD8^+^ CTLs into tumor tissues from combination-treated mice. a: control group; b: CCL21 treated group; c: anti-CD25 treated group; d: CCL21 combined with anti-CD25 treated group. Scale bar, 100 µm. (**B**) Flow cytometry analysis revealed that the combination treatment enhanced the frequency of effector cells at the tumor site, significantly more tumor-infiltrating CD4^+^, CD8^+^ T cells and CD11c^+^ DCs. *P < 0.05, **P < 0.01, compared with the control group. Similar results were obtained in three independent experiments.

### Evaluation of intratumoral cytokines production

To further evaluate the antitumor immune responses, intratumoral cytokines secretion after different treatments was detected by ELISA. Compared with the control and monotherapy groups, the combination treatment promoted significantly enhanced elaboration of IL-12 and IFN-γ, whereas revealed significantly reduced release of immunosuppressive mediators IL-10 and TGF-β1 (*P* < 0.01, Figure 7A–D).

**Figure 7:** Evaluation of intratumoral cytokines production after combination treatment. ELISA analysis for the intratumoral cytokine secretion profiles on day 7 after treatment initiation (n = 3 for each group). The combination treatment significantly enhanced the levels of IL-12 (**A**) and IFN-γ (**B**), but significantly reduced the levels of IL-10 (**C**) and TGF-β1 (**D**). *P < 0.05, **P < 0.01, compared with the control group. Similar results were obtained in three independent experiments.

## Discussion

The generation of an antitumor immune response is a complex process dependent on coordinate interaction of different subsets of effector cells, including both DCs and lymphocyte effectors. However, most tumors are not efficiently rejected despite their recognition by CD4^+^ and CD8^+^ T cells [29]. Tumor cells interfere with host DCs maturation, function and infiltration into the tumor [30,31]. Therefore, an implicit goal of immunotherapeutic approach designed to elicit an immune response against malignant cells is the migration of effector cells to the tumor site. It is believed that the most effective immunotherapies against solid tumors will be those that result in a large, sustained tumor infiltration by tumor-specific effector cells.

CCL21 can attract DCs and naive T cells to evoke effective antitumor immunity by binding to CCR7, which makes it a good therapeutic candidate against cancer. We have evaluated the antitumor responses in mice cancer models after administration of DCs genetically modified to express CCL21 [8,9]. More recent studies revealed a potential major role of Tregs in controlling the immune responses against tumors. It has been suggested that the presence of Tregs can explain the poor clinical efficacy of immunotherapeutic protocols in human tumors [32,33]. Although the precise mechanisms of suppression by Tregs remain to be determined, these cells can inhibit immune cell functions either directly through cell-cell contact or indirectly through the secretion of immunosuppressive mediators, such as IL-10 and TGF-β1 [18]. Hence, it is possible that by removing tumor-specific Tregs, antitumor immunity could be enhanced. Many studies in mice have shown that removal or inhibition of this subset of cells can enhance antitumor immune responses [34–37]. Accordingly, new immunotherapeutic strategies for tumors have increasely aimed at inhibition or depletion of Tregs. Depletion of Tregs by anti-CD25 mAbs could represent an important adjunct to cancer immunotherapy. However, solely depleting Tregs might not always result in tumor regression. Anti-CD25 mAbs will not only deplete Tregs, but also affect the effector cells expressing early activation marker CD25. Therefore, approaches combining Tregs depletion with other immunologic interventions might be more beneficial.

The recruitment or expansion of Tregs is closely correlated with early tumor growth [38]. Our findings also indicated that CD4^+^ CD25^+^ Foxp3^+^ Tregs gradually accumulated in the tumor tissue of mouse early-stage HCC. The presence of Tregs at the tumor sites emphasized their potential role to down-regulate the functions of effector T cell subsets. In this study, we investigated whether elimination of CD4^+^ CD25^+^ Tregs using anti-CD25 mAbs (PC61) was capable of enhancing CCL21-mediated antitumor immunity in a mouse HCC model. We showed that ip injection of anti-CD25 mAbs was capable of significantly eliminating CD25^+^ Foxp3^+^ Tregs within the tumor. Although anti-CD25 mAbs in the combination treatment group resulted in a proportion loss of activated CD25^+^ T cells, CCL21-mediated recruitment of T cells repaired and enhanced the effects of activated T cells. One resolution may be that the levels of CD25 appear higher and more stable on Tregs than activated effector cells. In addition, it is well documented that Tregs express higher levels of CD25 than activated T cells [39]. Nevertheless, the combination treatment with CCL21 and anti-CD25 mAbs maximally reduced CD25^+^ Foxp3^+^ Tregs from established tumors.

The results demonstrated that coadministration of CCL21 with anti-CD25 mAbs resulted in dynamic changes of CCR7 and Foxp3 expression, upregulation of CCR7 and inhibition of Foxp3 expression on day 1 to 7 after treatment initiation. The expression levels of two proteins were usually determined by the increased numbers of mature DCs and naive T cells and reduced number of Tregs within the tumor. In contrast to Tregs with a low CCR7 expression, mature DCs and naive T cells could be easily attracted to the tumor site by CCL21 due to their high CCR7 expression [14]. Tumor-associated DCs generally show an immature phenotype with low CCR7, which tends to induce immune tolerance and Tregs [20]. As a control, Foxp3 was markedly upregulated within the growing tumors, but CCR7 expression was inhibited at a low level. The results indicated that CCR7 expression inhibition might be associated with tumor poor immune status compared with Foxp3 expression increase in tumor progression. It should be noted here that CCR7 was not expressed on Hepal-6 cells (data not shown). Therefore, CCR7 could probably be acted as a prognosis for immunotherapies against tumors in our model. A variety of reports have indicated that, apart from chemotaxis, CCR7 controls the cytoarchitecture, the rate of endocytosis and the migratory speed of the DCs [40], also protects of circulating CD8^+^ T cells and DCs from apoptosis [41,42]. We have found that CCL21 contributes to the maturation of bone marrow-derived DCs (BMDCs), and strengthens their APC functions and induces secretion of IL-12 and IFN-γ [8]. In the present study, these findings supported and extended our previous studies demonstrating that the maturation of BMDCs stimulated by CCL21. Our current work is focused on the mechanism of CCL21 stimulating BMDCs maturation, the preliminary results suggest NF-κB signal may be involved in the process [43]. The functional axis encompassing CCL21/CCR7 makes up a key component in the initiation of the adaptive immune response. The interaction of DCs with CCL21 is essential for the function of these cells in tumor-bearing mice and may provide tools for novel therapeutic strategies.

We found that CCL21 in combination with anti-CD25 mAbs resulted in improved antitumor efficacy and prolonged survival, as well as blockade of tumor angiogenesis and cell proliferation. Apart from CCR7, mouse CCL21 also interacts with another receptor CXCR3, through which it can block angiogenesis in vivo [44]. Such bioactivity of CCL21 is conducive to induce antitumor immune responses. We believe that the inhibition of angiogenesis plays an important role in enhancing the antitumor effects of the combination treatment group. Further studies revealed that the combination treatment increased the frequency of tumor-specific CD4^+^, CD8^+^ T cells and CD11c^+^ DCs at the tumor site. Despite a small proportion loss of CD4^+^ T cells by anti-CD25 mAbs in the combination treatment group, there were significantly more tumor-infiltrating CD8^+^ CTLs and CD11c^+^ DCs. These data suggested that functional capacity of tumor-infiltrating effector cells was markedly enhanced after Tregs depletion in CCL21-treated mice, infiltration of activated CD4^+^ T cells and DCs in the Tregs-deprived tumor microenvironment might promote CD8^+^ T cells function, leading to effective T-cell priming and the generation of powerful antitumor immune responses. After combination treatment, the tumor site cellular infiltrates were accompanied by the enhanced elaboration of IL-12 and IFN-γ, but reduced release of the immunosuppressive mediators IL-10 and TGF-β1. IL-12 and IFN-γ mediate a range of biological effects that facilitate antitumor immunity [45], whereas IL-10 and TGF-β have been implicated in the induction or conversion of Tregs [46]. These results showed that the combination treatment was more effective in generating systemic antitumor responses.

It can be seen that CCL21-mediated antitumor response could be further boosted by depletion of Tregs. The precise mechanism involved in this process remains to be fully elucidated. We believe that CCL21 administration directionally attracts more mature DCs and naive T cells to the tumor site, ip injection of anti-CD25 mAbs both targets the suppressive activity of Tregs and reduces any risks of developing a systemic neutralizing antibody response [47].

In conclusion, our results demonstrated that in the Tregs-deprived tumor microenvironment, CCL21-mediated antitumor immunity was strongly improved, leading to a maximal therapeutic efficacy. The approach used here could also potentially be employed for an effective immunotherapeutic strategy against established tumors.
